This article has been retracted.

# Precision Strategy of Ideological and Political Education Using Big Data Analysis in Online Behavior Monitoring Environment

**DOI:** 10.1155/2022/2394668

**Published:** 2022-09-13

**Authors:** Yuefen Wang, Chaoqun Ma

**Affiliations:** School of Marxism, Northeast Forestry University, Harbin, Heilongjiang 150040, China

## Abstract

Ideological and political education (IPE) is aimed at achieving people's free and all-around growth through the use of appropriate methods, and the use of educational methods is integral to the execution of education. Under the influence of big data, it is imperative to strengthen the research on the accuracy of ideology education in colleges and universities (IPECU), which necessitates that ideology educators adopt big data thinking, investigate novel pedagogical approaches, and consistently develop new IPECU conditions. In this paper, a collaborative filtering- (CF-) based algorithm for IPE resource recommendations is presented. Users are given recommendations for educational resources based on their browsing history, browsing patterns, and preferences. The accurate recommendation system can determine users' needs by examining how they use the website in order to suggest more useful information to them. In comparison to the conventional algorithm, the accuracy of the ideological and political education precision recommendation model in this study is 16.75% greater. Teachers can use big data technology to gather students' data information that is dispersed throughout cyberspace, understand students' states in real time, and deliver accurate instructional materials in accordance with students' various states and needs by utilizing the intelligent ideology mode.

## 1. Introduction

The Internet industry has driven the development of a number of other traditional industries while its rapid development and traditional industries have embraced the Internet across borders. The cross-border of the education industry is also quietly going on. It is imperative to effectively combine the value logic of the education industry with the operation logic of the Internet industry [1]. The purpose of IPE is to use appropriate methods to achieve people's free and all-round development, and the implementation of education cannot be separated from the application of educational methods. IPE methods are the key to the implementation of IPE, which restricts the effectiveness and development of IPE to a certain extent [2]. With the advancement of IT, networks have permeated many facets of social life. In particular, network teaching has resulted from the widespread use of IT in higher education. Although many institutions have adopted online instruction in IPE, the development of online instruction for Ideology courses is constrained by the insufficient design of online instructional resources [3]. The accuracy of IPECU research must be strengthened in the big data era, which necessitates that ideology educators adopt big data concepts, experiment with new teaching techniques, maintain a tight relationship with reality, life, and students, and continually develop new IPECU scenarios [4].

The Internet industry has driven the development of a number of other traditional industries while its rapid development and traditional industries have embraced the Internet across borders. The cross-border of the education industry is also quietly going on, and it is imperative to effectively combine the value logic of the education industry with the operation logic of the Internet industry [5, 6]. With the widespread use of precision technology, the recommendation system has gradually become the focus of attention and research, because it actively recommends resources to customers to meet user needs. Many users are unwilling to spend too much time on a website that takes a long time to find resources. With the advent of the age of big data, it is a strategic choice for IPE in the age of big data to drive high-end IT and transform the paradigm of intelligent IPE, so that intelligent IPE presents a brand-new development trend. The rapid development of education is reshaping educational concepts, innovating educational contents and methods, and accelerating the reconstruction of educational ecology. Therefore, the construction of wisdom and ideological education has become an inevitable choice for the reform and innovation of IPE. Big data IT can provide support for the precise reform of IPECU, help IPECU comprehensively and systematically analyze the information of the subject and object of education, accurately identify the learning needs of educational objects, accurately evaluate the effect of education, accurately push educational resources, accurately match the educational needs and educational supply for IPECU, and drive the IPECU to achieve accurate reform [7]. This paper proposes a recommendation algorithm of IPE resources based on CF algorithm. According to users' browsing records, browsing habits, and preferences, the instructional resources that users may be interested in are recommended to users. Through design experiments, the effectiveness of the algorithm is proved.

Under the influence of big data thinking, the essence of education gradually returns to promoting the individual development of learners. Educators use big data to analyze all the digital records of learners' learning behaviors in order to improve the teaching process and enhance the learning effect. The construction of network instructional resources is very important for the development of network teaching of IPECU. Without rich and complete network instructional resources, network teaching of Ideology courses in Universities will be impossible [8, 9]. As an important way to guide students to form correct values, IPE must be combined with big data to realize the accuracy of IPECU and guide the formation of correct values of educational objects, which is also an important responsibility and mission of the school and even the society. Applying big data technology and concept to the practice of IPECU has not only great theoretical significance but also important practical significance. For the precise strategy of IPE resources, the main innovations of this paper are as follows:

1. By analyzing users' behavior in the website, the precise recommendation system can infer users' needs, so as to recommend more valuable resources to users. The recommendation quality of the recommendation system directly determines the user's dependence on the recommendation system
2. This paper is aimed at designing and implementing a precise learning resource recommendation strategy based on CF algorithm. According to the user's browsing records, browsing habits, and preferences, the instructional resources that users may be interested in are recommended to users, and the CF algorithm is used to recommend precise chemistry learning resources for learners

The rest of the chapters are arranged as follows: the second section is related work, which analyzes the research of excellent scholars in IPE and teaching recommendation; the third section constructs the IPE resource recommendation model of this paper; the fourth section verifies the effectiveness of the model through experiments; the fifth section summarizes the contribution of this paper and puts forward that in the future, it is also necessary to refine the description of the data entities of learning resources, such as the course category of learning resources and the applicable population.

## 2. Related Work

### 2.1. Big Data and Ideology Teaching

The focus of education increasingly shifts back to supporting students' individual growth under the influence of big data thinking. Big data is used by educators to analyze all of the digital records of students' learning behaviors in an effort to optimize teaching and learning outcomes. Big data, according to Ym et al., has given us a fresh outlook and a fresh way to understand the world, and it has sparked the reform of IPE methodology [10]. Toledo and Mota emphasised that the current integration of educational resources in IPE suffers from the phenomena of blind resource accumulation, complex resource structure, and dated resource content. The development of college students' moral, intellectual, and skill levels has evolved into the target direction for the integration of online learning resources in IPE, guided by IPE theory [11]. In view of the practical problems faced by the current network teaching of IPECU, Chen et al. promote the network teaching of IPE by improving the construction of network instructional resources [12]. Cakir and Simsek think that students' satisfaction with the utilization rate of online instructional resources is low, and they hold a positive attitude towards the necessity of setting up the IPE instructional resource network but think that there are big problems in the website at present [13]. Therefore, we should further optimize the ideology course instructional resource network, enrich its content, innovate its forms of expression, and enhance its interaction, so as to assist the ideology course teaching and improve its timeliness.

### 2.2. Teaching Recommendation Algorithm

With the rise of big data, the traditional IPE methods are bound to undergo fundamental changes. Using data, we can more comprehensively analyze, grasp, and predict the changes of students' thoughts and behaviors and create a new research model of IPE. Koren generated the user model through the history of the user's purchase and made recommendations according to the user model [14]. Pang et al. suggested that logs can be mined to help improve the accuracy of recommendation system [15]. Pan et al. and Li et al. used decision tree technology, mining, association rule mining, and e-commerce recommendation systems to recommend things that would be useful to customers [16, 17]. According to students' interests and progress, Zhang et al. and Bobadilla et al. suggested a system for proposing current and upcoming learning resources in real time [18, 19].

The research on the recommendation system of educational resources is not very mature. Because the popularity of teaching assistant system in domestic education is not very high, although some universities have their own teaching assistant systems, these teaching assistant systems rarely contain instructional resource recommendation subsystems. Deeply cultivating big data in the field of IPECU and promoting the construction of a set of intelligent ideology mode with complete system, coupled elements, coordinated development, and efficient operation will continuously improve and deepen the knowledge system and theoretical foundation of IPECU.

## 3. Methodology

### 3.1. CF Recommendation Algorithm

The enormous potential of the network can connect thousands of computers, mobilize people from different regions and different responsibilities to work together, and allow people from different regions to communicate with each other. Big data provides a new research paradigm and a new thinking paradigm for the research of IPECU, promotes the scientific construction of IPE, and makes accurate IPE possible. Content-based recommendation technology takes resource information as the research object, uses information retrieval technology to analyze the content of items, and usually applies neighbor function and classification technology to analyze and cluster the text content of items. Content-based recommendation method needs to establish documents for each user's access content, and at the same time, classify the contents of websites, such as commodities in business websites, course contents in educational websites, etc. When users visit this website, documents should be made according to the user's access content. The enormous potential of the network can connect thousands of computers, mobilize people from different regions and different responsibilities to work together, and allow people from different regions to communicate with each other.

When a new user operates, the algorithm will train its neural network according to the user's operation, so as to achieve accurate recommendation. By copying the global recommendation model as the recommendation model of the new user, and then modifying the recommendation model according to the subsequent operations of the new user, the recommendation model is closer to the user's preference. Views of this process are shown in Figure 1.

Let *C* be the set of all users, and *S* be the set of all recommended objects. Generally speaking, the scale of the collection *C* and the collection *S* is relatively large, such as millions of online customers and hundreds of millions of commodities. Calculating the recommended object, for the recommendation degree of user *C*, we use the recommended utility function *u*(*c*, *s*), that is, *u* : *C*∗*S* − *R*, and *R* is a nonnegative real number; the problem to be studied by the recommendation algorithm becomes to find the set *S*^∗^ of those recommended objects with the largest recommendation degree *R*:

(1) $$\begin{array}{c} \forall c\in C,S^{*}=\arg\max_{s\in S}u\left(c,s\right). \end{array}$$

According to actual problems, different attribute feature information can be used when measuring and sampling users or recommended objects. Calculating the utility value *u* is the core problem of the recommendation algorithm, but it is not in the whole field of *C*∗*S*, but distributed in a subspace. For a certain data set, the *u* should be extrapolated first, that is, the recommended objects should be marked with the user's historical rating, and the recommended objects that have not been evaluated by the user need to be marked and extrapolated before use. Various recommendation algorithms have designed corresponding utility functions for different extrapolation and prediction strategies.

The advantage of using content-based method for accurate recommendation is simple and effective. However, there are still some problems [20]. Content-based methods need to do a lot of analysis work before recommendation, such as what the current users visit and which pages in the website are related to it. Big data IT can provide support for the precise reform of IPECU, help IPECU comprehensively and systematically analyze the information of the subject and object of education, accurately identify the learning needs of educational objects, accurately evaluate the effect of education, accurately push educational resources, accurately match the educational needs and educational supply for IPECU, and drive the IPECU to achieve accurate reform. According to these data, the system can make accurate recommendations.

Let the number of documents contained in the document set be *N*, the number of documents containing the keyword *k*_*i*_ in the document set is *n*_*i*_, *f*_*ij*_ represents the number of times the keyword *k*_*i*_ appears in the document *d*_*j*_, and the word frequency *k*_*i*_ of *d*_*j*_ in the document TF_*ij*_ is defined as

(2) $$\begin{array}{c} {\text{TF}}_{ij}=\frac{f_{ij}}{\max{zf}_{zj}}, \end{array}$$

where *z* represents the keyword appearing in the document *d*_*j*_. The inverse frequency IDF that *k*_*i*_ appears in the documentation set is defined as

(3) $$\begin{array}{c} \text{IDF}=\log\left(\frac{N}{n_{i}}\right), \end{array}$$

where *n*_*i*_ represents the number of documents that contain keywords in the document. The importance *W*_*ij*_ of the keyword *k*_*i*_ in the document *d*_*j*_ is defined as

(4) $$\begin{array}{c} W_{ij}={\text{TF}}_{ij}*\text{IDF}. \end{array}$$

Assuming that the similarity between items *S* and *U* is calculated, the algorithm obtains the importance of the keyword *k*_*i*_ in the document *d*_*j*_ and then sorts the importance *W*_*ij*_ of all words in descending order to obtain the real keyword of the item. Assume that the keywords with the word frequency value ranking in the top *N* are selected.

The user's interest in a given thing can be anticipated by assessing how closely an item and the user's interest traits resemble one another. Typically, the cosine similarity method is employed to assess how similar they are:

(5) $$\begin{array}{c} \text{sim}\left(u,v\right)=\frac{u\cdot v}{\left|u\right|\left|v\right|}. \end{array}$$

Vectors *u* and *v* can represent user interest model vector and commodity feature vector, respectively. If the sim(*u*, *v*) value is larger, the similarity between the two is higher, and vice versa.

The decision to drive high-end IT and change the paradigm of intelligent IPE in the age of big data, where intelligent IPE presents a brand-new development trend, is one made strategically by IPE. Education is rapidly evolving, which is altering educational concepts, developing educational materials, and hastening the reconstruction of educational ecosystem. As a result, the development of wisdom and ideological education has emerged as an unavoidable option for IPE's reform and innovation. The user's access records within a particular amount of time are the most effective for users, and if it takes too long, the things accessed earlier may not be the content that users are interested in [21]. This means that while evaluating users' interests, we also need to take time into account. Focusing on the dimension of wisdom education, this paper holds that wisdom and ideological education is a new form of wisdom education in the field of IPE. In the construction of intelligent education environment, the construction of intelligent ideology cloud needs to be built and improved, so as to serve teaching monitoring, online teaching, psychological counseling, resource supply, instant feedback and so on. Content-based filtering recommendation algorithm combines the data provided by information retrieval to screen information and finally achieves the purpose of recommending items to users.

In the similarity calculation of CF algorithm, two user variables or two item variables need to be extracted from the system. When the numerical changes of the two variables are positively correlated, it means that the two variables have a linear relationship, and the similarity between users or projects is high. When the values of the two variables change into negative correlation, it means that the two variables have no linear relationship, and the similarity between users or projects is low. The calculation formula of Pearson coefficient is:

(6) $$\begin{array}{c} \rho_{x,y}=\frac{\sum xy-\left(\sum x\sum y/N\right)}{\sqrt{\left(\sum x^{2}-\left({\left(\sum x\right)}^{2}/N\right)\right)\left(\sum y^{2}-\left({\left(\sum y\right)}^{2}/N\right)\right)}}. \end{array}$$

When the Pearson coefficient is applied in the user-based CF algorithm, the calculation formula of the Pearson coefficient will make a relative change, and the similarity calculation formula is as follows:

(7) $$\begin{array}{c} \omega \left(u,v\right)=\frac{\sum_{i\in 1\left(u\right)\cap 1\left(v\right)}\left(r_{ui}-{\bar{r}}_{u}\right)*\left(r_{vi}-{\bar{r}}_{v}\right)}{\sqrt{\sum_{i\in l\left(u\right)\cap l\left(v\right)}{\left(r_{ui}-{\bar{r}}_{u}\right)}^{2}}\sqrt{\sum_{i\in 1\left(u\right)\cap l\left(v\right)}{\left(r_{vi}-{\bar{r}}_{v}\right)}^{2}}}. \end{array}$$

where *ω*(*u*, *v*) is the similarity calculated by user *u* and user *v* based on the Pearson coefficient.

*I*(*u*) is the set of items reviewed by user *u*, and *I*(*v*) is the set of items reviewed by user *v*. *r*_*ui*_ is user *u*'s preference for item *i*, and *r*_*vi*_ is user *v*'s preference for item *i*. ${\bar{r}}_{u}$ and ${\bar{r}}_{v}$ represent the average level of preference value of user *u* and user *v* on all items, respectively.

With the help of high-end IT such as big data, the construction of IPE will realize digitalization, integration of things and intelligence of IPE. This will fundamentally change the traditional mode of IPE, break through the limitations of the original mode of single subject education, and realize the cooperative education of all staff. Compared with the traditional IPE model, the intelligent IPE model highlights the concept of collaborative education and strives to build an intelligent IPE resource database, including instructional resource database, user behavior database, and educational administration information management database, to provide intelligent services for all educational subjects and to form an educational joint force of multilinkage, multiforce, and multichannel progress.

### 3.2. Precise Recommendation of IPE Instructional Resources

Users of the instructional resource sharing module are mainly divided into student users and teacher users. Students and teachers can not only browse, search by category, search by keyword, upload and download the resources but also rate and comment on the resources, so as to realize the reasonable positioning of the resources' value. The instructional resource precision recommendation module is mainly aimed at student users. The recommendation system includes three parts: keyword layer, description layer, and user interface layer. At the bottom of the keyword layer, it provides the required keywords for the upper description and defines the dependencies between keywords. The description layer above the keyword layer defines the description of users and resources. At the top user interface layer, according to the precise rules defined in the following two layers, resources satisfying the rules are recommended to users. The recommendation method of IPE instructional resources based on CF is shown in Figure 2.

In the era of big data, intelligent IPECU is the unavoidable trend of precise IPECU. Teachers gather a large amount of information about educators' educational practices with the aid of big data technology [22]. At the same time, the corresponding *α* and *β* should be set according to the contribution degree of the weighted mean score of users and the weighted mean score of items. Wherein, the weighted mean score of user *i* is calculated:

(8) $$\begin{array}{c} r_{u}={\bar{r}}_{u}+\frac{\sqrt{\sum_{k=1}^{k}{\left(r_{k,i}-{\bar{r}}_{i}\right)}^{2}}}{K}. \end{array}$$

In the formula, *K* is the total number of user ratings for item *i*, and *r*_*u*,*q*_ is the rating value of user *k* for unrated item *i*. The user's weighted mean rating is the sum of the mean errors of the user's average rating *r*_*u*_ and the user's various ratings ${\bar{r}}_{u}$ relative to the average rating of the unrated items. Calculate the weighted mean score for *i* items:

(9) $$\begin{array}{c} r_{i}={\bar{r}}_{i}+\frac{\sqrt{\sum_{q=1}^{Q}{\left(r_{u,q}-{\bar{r}}_{i}\right)}^{2}}}{Q}, \end{array}$$

where *Q* is the total score of user *u* to the project space and *r*_*u*,*q*_ is the score value of *k* to user *u* and to *q*. The weighted mean rating of an item *r*_*i*_ is the sum of the average rating of the item ${\bar{r}}_{i}$ and the mean error of the average rating of each user in the user set for the unrated item *i* and the average rating of the user. Then integrate the weighted score:

(10) $$\begin{array}{c} r_{ui}={ar}_{u}+\beta ri\;\alpha +\beta =1. \end{array}$$

Any item in the matrix has a score for the items *i* and *j* after collecting the integrated weighted score of the unscored items and filling the corresponding items, and the contribution judgement parameters *α* and *β* are introduced.

Although precise learning is also mentioned in the traditional education model, students' learning tends to keep a unified pace due to the constraints of scientific and technological level, ideas, and other factors. To some extent, learning in the Internet is naturally characterized by precision. Learners can break through the time and space constraints and freely choose learning content, teachers, etc., in the open online learning space and shared intelligent learning platform, which has great autonomy and freedom. However, without the support of big data, teachers cannot dig out the teaching rules hidden behind it through educational big data, nor can they accurately identify learners' precision needs. The intelligent teaching system automatically generates feedback reports for each learner based on accurate evaluation, gives accurate learning suggestions, and pushes them to learners. Students can accurately orient and exert their strength, aim at the short board, target treatment, and make breakthroughs. IPE will collect and record educational data in real time through various mobile internet application platforms, with the help of relevant IT, and conduct in-depth mining, classification and processing, so as to deeply analyze the correlation between data and obtain accurate feedback. This can not only help ideology educators to deeply understand the objective laws of teaching management but also help ideology educators to accurately grasp the “whole portrait” of students' groups in terms of ideological state, behavior dynamics, and knowledge mastery and provide data reference for the next teaching management.

## 4. Result Analysis and Discussion

Make data education decision-makers' decision-making more scientific, and information technology becomes a key reference point for decision-making. In line with the overall trend, opportunities and problems are interlaced while the drawbacks of conventional IPE procedures become more pronounced. The emergence of drawbacks is a crucial element in fostering further IPE method innovation. Through the real-time collection and in-depth analysis of data, instructors can digitally record particular behavior data from students' lives, track mental changes in their students, shape their personalities, and implement focused education through minor behaviors. The informationization offered by big data can help the educated understand the macrolevel trends in student development. On the basis of evaluating and understanding students' ideas and actions, educators may more accurately forecast the growth trend of students' thoughts and behaviors in the educational setting. Big data analysis can help advance the combination of precise development and mass customization by clearly revealing the ideological context of student groups and individuals and by grasping the behavioral traits of these groups and individuals. The findings of users' subjective evaluations of various suggested models of IPE instructional resources are displayed in Figure 3.

The majority of users reported that the precise recommendation system of learning resources can assist them in quickly locating the information they need among the vast learning resources, and the results of the recommendations are typically more accurate, which can meet individual needs and tap into users' potential interests. When different levels of sparsity are chosen, the algorithms' performance is compared in Figure 4.

From the form of collecting and using information data of big data platform, when collecting information resources of IPE, universities should comprehensively include teachers, college students, counselors, and other subjects involved in IPE activities and comprehensively collect and sort out relevant data of their participation in education.  Table 1 shows the change of model accuracy when different iterations are set. Six groups of data with iteration times between 2000 and 12000 were selected to observe the change of model accuracy.

It is clear that over numerous rounds, the algorithm's accuracy progressively increases and starts to stabilise. Teachers must learn to use data to analyze and solve problems, truly comprehend the benefits of using big data, and lead the use of big data technology with appropriate data governance ideas in order to achieve the perfect transformation of IPE with the aid of big data technology.  Figure 5 displays the MAE outcomes for the various algorithms.  Figure 6 displays the recall of several algorithms.

Table 2 shows the experimental results of screening evaluation indexes. Comparison of recommended accuracy between models is shown in Figure 7.

It is not difficult to see that the recommendation algorithm in this paper has a high accuracy, which is 16.75% higher than the traditional recommendation algorithm. The users' evaluation of the accuracy of the recommendation results of the learning resource precision recommendation system is scattered. The construction of network instructional resources of IPECU can greatly promote the network teaching of IPECU. Its in-depth development can realize the sharing of network instructional resources of IPE, enrich the content of network teaching of IPECU, stimulate students' learning enthusiasm, and improve the effect of network teaching of IPECU. A large part of the reason lies in the fact that there are not many users and resources in the system at the early stage of transportation. Most of the recommendations can only be made according to the user-resource label, and the CF algorithm fails to exert its real evaluation ability. When the number of users and resources on the system reaches a certain number, the recommended results will be more accurate.

## 5. Conclusions

Although many institutions have adopted online education in IPE, the development of online instruction for courses in ideology is constrained by the subpar design of online learning tools. The development of IPECU's network instructional tools can significantly advance network instruction at the university. Its thorough development can make it possible to share network instructional resources from IPE, enrich the curriculum of network instruction from IPECU, pique students' interest in learning, and enhance the impact of network instruction from IPECU. The CF algorithm is employed in this paper to analyze user preferences. The instructional resources that users may be interested in are recommended to users based on their browsing history, browsing patterns, and browsing preferences, and the CF algorithm is used to recommend specific learning resources for students. The findings indicate that this model's suggestion accuracy is 16.75% more than that of the conventional recommendation algorithm. Teachers can use big data technology to collect students' data information that is dispersed throughout cyberspace, understand students' states in real time, provide accurate instructional resources, and create specialised lesson plans based on the needs and states of their various students by utilizing the exploration of intelligent ideology mode.

## Figures and Tables

**Figure 1:** Precise recommendation process.

**Figure 2:** Recommendation method of instructional resources for IPE.

**Figure 3:** User subjective rating.

**Figure 4:** Performance comparison between algorithms with different sparsity.

**Figure 5:** Mean absolute error results of different algorithms.

**Figure 6:** Recall results of different algorithms.

**Figure 7:** Recommendation accuracy results of different models.

**Table 1:** Model accuracy with different iterations.

Iterations	Accuracy rate
2000	32.6%-67.5%
4000	43.4%-71.8%
6000	61.2%-73.5%
8000	71.4%-85.6%
10000	80.3%-92.3%
12000	81.2%-93.6%

**Table 2:** Experimental results of filtering evaluation indicators.

Model	Average precision	Average recall
Weighted association rules	88.35%	90.41%
Literature [17] algorithm	83.14%	85.31%
Paper recommends model	94.25%	95.18%

## Data Availability

The data used to support the findings of this study are available from the corresponding author upon request.
